# The Predictive Value of Changes in the Absolute Counts of Peripheral Lymphocyte Subsets for Progression and Prognosis in Breast Cancer Patients

**DOI:** 10.1155/2022/3444360

**Published:** 2022-08-18

**Authors:** Aqing Liu, Ying Xia, Wentao Li, Guan Zhang, Yunhe Liu, Songshan Ye, Zhijie-ruo Zhao, Yanjie Yang, Yingjie Jia, Yongtie Guo, Xu Liu, Huayu Chen, Jianchun Yu

**Affiliations:** ^1^Department of Oncology, First Teaching Hospital of Tianjin University of Traditional Chinese Medicine, National Clinical Research Center for Chinese Medicine Acupuncture and Moxibustion, Tianjin, China; ^2^Graduate School, Tianjin University of Traditional Chinese Medicine, Tianjin, China; ^3^Clinical Laboratory, First Teaching Hospital of Tianjin University of Traditional Chinese Medicine, Tianjin, China

## Abstract

**Background:**

As the number and proportion of lymphocyte subsets are an important indicator of the immune function, an in depth understanding of the immune function of patients with malignant tumor has important clinical values for the treatment, prognosis, and evaluation of the disease. This retrospective study was to evaluate the clinical value of the absolute counts of lymphocyte subsets as potential blood biomarkers for progression and prognosis in breast cancer patients.

**Methods:**

A total of 237 BC patients and 55 age-matched female normal healthy donors were included in this study. Flow cytometry was used to determine the absolute counts and the percentages of CD3^+^, CD4^+^, CD8^+^, B, and NK cells. The receiver operating characteristic curve (ROC) was used to evaluate the accuracy of absolute count of lymphocyte subsets in the curative efficacy assessment. The clinicopathological parameters influencing the disease progression were determined by Cox proportional hazards regression. Progression-free survival (PFS) was estimated using the Kaplan–Meier method with the log-rank test. Results: Compared with the healthy donors, the absolute counts of lymphocyte subsets in patients decreased significantly. ROC analysis showed that the area under the curve of the CD4^+^ absolute count was 90% (95% confidence interval 0.859–0.940), and the sensitivity and specificity were 80.9% and 85.3%, respectively. The analysis of Cox regression showed that the cutoff value of the CD4^+^ absolute count ≥451 cells/*μ*L might be a favorable prognostic factor. Multivariate analysis of prognostic factors of PFS showed that the CD4^+^ and CD8^+^ absolute count were independent factors for predicting PFS.

**Conclusions:**

The remarkably impaired absolute counts of the CD3^+^, CD4^+^, CD8^+^, B, and NK cells in patients with breast cancer can be used as potential susceptible biomarkers to evaluate the patient's immune status. The higher level of CD4^+^ and CD8^+^ absolute counts probably contributed to the longer PFS and favorable outcome of BC patients.

## 1. Introduction

Breast cancer (BC) has become one of the main causes of cancer death in women worldwide. According to the latest statistics in 2020, with an estimated 2.3 million new BC cases and 685,000 deaths caused by BC [1], the number of BC patients in 185 countries and regions has overtaken that of lung cancer patients, and BC becomes the most commonly diagnosed cancer. In recent years, the incidence rate of BC has been increasing, and the age of its victims has been getting younger [2]. At present, the main treatments of BC are surgery, chemotherapy, endocrine, and other comprehensive therapies. For patients with early and mid-term BC, postoperative adjuvant chemotherapy can improve the local control rate and reduce the recurrence rate of local and regional lymph nodes [3].

It has been found that the recurrence and metastasis of tumors are closely related to the decline of the immune function, which in turn leads to the tumor immune escape [4]. The classical lymphocyte subsets include CD3^+^, CD4^+^, CD8^+^, B, and natural killer (NK) cells, which are essential for regulating the immunity and specific killing of tumor cells [5]. Although their compositions are simple, their roles in immune responses are diversified, including both innate and adaptive immunity, and cellular and humoral immunity as well. The CD4^+^ can activate other lymphocyte subsets by releasing cytokines and suppress tumor development by directly killing tumor cells that express adequate levels of major histocompatibility complex (MHC) class II molecules [6]. The CD8^+^ cells, a kind of cytotoxic cells, can recognize tumor cells that express MHC class I molecules presented by antigen-presenting cells and produce IFN-*γ*, perforin, and granzyme B for targeting and killing tumor cells [7]. B cells play an important role in the humoral immunity, which not only can present antigens to T cells and participate in the immune response of T cells but also can recognize different antigen epitopes, secrete immunoglobulin, and participate in the humoral immune response [8]. NK cells, as indispensable effector cells in the innate immune system, work as the first line of defense for the host immune defense against cancer and pathogens [9]. Therefore, analyzing peripheral lymphocyte subsets is a significant and convenient way to assess the immune function, which includes the percentages of lymphocytes (PL) and the absolute count of lymphocytes (ACL). In particular, the ratio of the CD4^+^ to CD8^+^ may indicate the balance of the immune system, which is maintained by the proportion and the number of peripheral blood lymphocytes [10]. Growing evidence has revealed the absolute count of peripheral blood lymphocyte subsets is positively correlated with the prognosis of cancer patients [11–13].

Traditionally, the ACL was measured by the dual-platform technology, which combined the percentage of lymphocyte subsets assessed by flow cytometry with the absolute lymphocyte count assessed by an automatic hematology analyzer. However, this method produced obvious discrepancies among different laboratories [14–17]. Herein, we adopted a single-platform technology to carry out the detection entirely on flow cytometer. This method significantly improved the accuracy of the analysis. Previous studies showed that lymphopenia, or low peripheral blood lymphocyte count, can predict higher mortality and increased risk of recurrence after primary surgery and neoadjuvant therapy, whereas higher absolute lymphocyte counts can predict lower mortality from early-stage triple-negative BC [18, 19]. Nevertheless, these studies only analyzed the total number of lymphocytes but did not further analyze the influence of the ACL on the immune function. As a result, the correlations between prognosis and the ACL in BC patients remain unclear.

This study aimed at evaluating the predictive value of PL and ACL for BC progression and prognosis, and analyzing the importance and susceptibility of ACL used as biomarkers of immune impairment.

## 2. Methods

### 2.1. Clinical Data

A total of 237 BC patients and 55 age-matched female normal healthy donors [normal controls (NCs)] were enrolled in the First Teaching Hospital of Tianjin University of Traditional Chinese Medicine, Tianjin, China, from January 1, 2018 to October 31, 2020. The cohort of 237 patients were all women with a median age of 64 years (ranging from 36 to 80 years), including 208 postmenopausal patients and 29 premenopausal patients. NCs were all females with a median age of 64 years (ranging from 35 to 80 years), including 7 premenopausal females and 48 postmenopausal females. No significant difference was found in the age and menstrual status between the two groups (*P* > 0.05). All the subjects were given the informed consent in accordance with the Declaration of Helsinki, and the clinical trial was approved by the hospital ethics committee (TYLL2017[K]002, 25 December 2017) and registered at Chinese Clinic Trial Registry (ChiCTR-IOR-17014139).

### 2.2. Inclusion Criteria

#### 2.2.1. BC Patients

Inclusion criteria were as follows: (1) pathologically ascertained diagnosis of malignant BC and disease stages determined according to the tumor-node-metastasis (TNM) classification scheme recommended by the Union for International *Cancer* Control, (2) at least one measurable lesion according to the Response Evaluation Criteria in Solid Tumor (RECIST) (version 1.1) (20), (3) without other malignant tumors, (4) a baseline Eastern Cooperative Oncology Group (ECOG) performance-status score of 0 or 1, and their expected survival ≥6 months, (5) complete clinical and laboratory data including PL and ACL, and (6) no underlying conditions such as severe hypertension, diabetes, coronary heart disease, infectious diseases, hematopoietic system, and immune system diseases.

#### 2.2.2. NCs

Subjects who served as NCs were inquired about their physical condition, medication, smoking, and alcohol consumption. The NCs, showing normal blood routine examination, liver functions (AST and ALT), renal functions (SCr), blood glucose levels, and without tumors, were considered normal.

### 2.3. Exclusion Criteria

#### 2.3.1. BC Patients

Exclusion criteria were as follows: (1) undetermined diagnosis of breast malignancy; (2) other malignant tumors; (3) difficulty with tracing their personal data and clinical case data; (4) underlying conditions such as acute infection, hematological disorders, autoimmune diseases, pregnancy, or lactation; and (5) not following medical advice.

#### 2.3.2. NCs

Healthy physical examinees with breast disease, immune system diseases, metabolic diseases, acute infection, or tumors were excluded.

### 2.4. Treatments

All the subjects underwent the following treatments. (1) Surgery: 83 patients received no other treatments except surgery, including mastectomy or lumpectomy with sentinel node biopsy or full axillary dissection. (2) Surgery combined with chemotherapy: 82 patients received postoperative chemotherapy, including neoadjuvant/adjuvant chemotherapy within one year of diagnosis. The treatment regimens employed were paclitaxel/epirubicin/cyclophosphamide/docetaxel (CE/TAC). (3) Surgery combined with endocrinotherapy: 72 patients received postoperative endocrinotherapy. The endocrine therapy for premenopausal BC patients with positive estrogen/progesterone receptor (ER/PR) was dominated by tamoxifen, whereas the endocrine therapy for the postmenopausal patients with positive ER/PR was dominated by letrozole.

### 2.5. Efficacy Evaluation

Based on RECIST (version 1.1) [20], the efficacy evaluation was divided into complete response (CR), partial response (PR), stable disease (SD), and progress disease (PD). CR + PR was considered to be the response (*R*) group, whereas SD + PD was considered the nonresponse (NR) group.

### 2.6. The Main Reagents and Instruments

Lymphocyte subsets were assayed by using a lyse/no-wash procedure based on a single-platform technique of ten-color flow cytometry (BD FACS Canto II : U6573380-00541, USA). The reagents were BD Multitest IMK kit (catalog no.: 662965) containing BD Multitest CD3FITC/CD8PE/CD45PerCP/CD4APC and BD Multitest CD3 FITC/CD16^+^CD56^+^PE/CD45PerCP/CD19APC, and BD Multitest IMK kit lysing solution (catalog no.: 91–1087). The EDTA blood collecting tubes and trucount tubes (catalog no.: 340334) were also purchased from BD Biosciences, USA.

### 2.7. Sample Collection

Two milliliters of fresh whole blood drawn from the NCs and BC patients were stored in the EDTA-anticoagulant blood collecting tubes.

### 2.8. Cellular Staining and Analyzing

Whole blood of the 292 participants was collected and assayed by flow cytometry following the BD operating instruction. In brief, for each sample, two trucount tubes were labeled with letters A and B to distinguish them from each other. 20 *μ*L of BD Multitest CD3^+^/CD4^+^/CD8^+^/CD45^+^ and CD3^−^/CD16^+^CD56^+^/CD45^+^/CD19^+^ reagents was added to the bottom of tubes A and B, respectively. Then, 50 *μ*L of well-mixed whole blood was added to the bottom of every tube. Finally, 450 *μ*L of lysing solution was added into every tube, mixed, and incubated for 15 min in dark at room temperature for analysis.

### 2.9. Statistical Analysis

The normality of statistical data was evaluated by the Shapiro–Wilk test, using two independent sample *t*-tests to analyze the differences in PL and ACL between BC patients and NCs. The differences among three or more groups of continuous numerical variables with normal distribution were analyzed by one-way ANOVA (the Bonferroni test or the Tamhane test). Progression-free survival (PFS) was defined as the time from the date of enrollment to disease progression, recurrence, or death. The follow-up deadline was 31 January 2021. The receiver operating characteristic curve (ROC) was used to evaluate the accuracy of ACL in the curative efficacy assessment. Categorical variables were analyzed using the chi-squared test. Survival curves were constructed using the Kaplan–Meier method. Univariate and multivariate Cox proportional hazards regression analyses were performed to assess the relationship between clinicopathological parameters and PFS. Variables with a *P* value < 0.05 by a univariable analysis were entered for multivariable analysis. Hazard ratio (HR) was reported with 95% confidence interval (CI). All tests were 2-tailed and *P* < 0.05 was considered statistically significant. The data were analyzed by SPSS 25.0 (IBM Corporation, USA). Figures were prepared using GraphPad Prism software (version 9.0) (San Diego, USA).

## 3. Results

### 3.1. Patient Characteristics

The clinicopathological features of 237 BC patients are described in Table 1. Among these BC patients, 148 (63.4%) were diagnosed with stage III–IV disease, 181 (76.4%) were medium/low differentiation, 158 (66.7%) had lymph node metastasis, 117 (49.4%) had distant metastasis, and 116 (48.9%) had family history. A total of 209 (88.2%) patients were diagnosed with invasive ductal carcinoma (IDC), while 28 (11.8%) patients were diagnosed with invasive lobular carcinomas (ILC).

### 3.2. Comparison of ACL between BC Patients and NCs

To investigate the changes in the ACL of BC patients, we compared the ACL of BC patients and NCs. The results showed that there was no difference in the percentages of ACL between the two groups (*P* > 0.05) (Figure 1(a)). However, compared to NCs, the absolute counts (AC) of CD3^+^(929.03 ± 241.42 vs. 1680.24 ± 549.30), CD4^+^(442.58 ± 97.05 vs. 933.60 ± 340.92), CD8^+^ (321.49 ± 112.56 vs. 647.42 ± 280.40), B (178.44 ± 80.43 vs. 283.35 ± 157.74), and NK (174.54 ± 71.44 vs. 400.04 ± 162.08) cells were decreased significantly in BC patients (*P* < 0.001) (Figure 1(b)). These results suggested that it was ACL rather than PL that decreased in BC patients. To our knowledge, PL represents the proportion or composition of each subset, revealing the development and differentiation of lymphocytes, whereas the ACL demonstrates the exact number of peripheral lymphocyte subsets, revealing the proliferation of lymphocyte progenitor cells. These results indicated that the proliferating ability of lymphocytes was impaired noticeably in BC patients.

In addition, the PL in BC patients at stages I-II and III-IV, compared with that in NCs, showed no significant difference (*P* > 0.05) (Figures 1(c) and 1(e)), whereas significant differences between the two groups were observed in their ACL (*P* < 0.001) (Figures 1(d) and 1(f)). These results suggested that a significant decrease in the ACL was characteristic of immune impairment or a sign of immunodepletion in BC patients.

### 3.3. ACL in BC Patients at Different Clinical Stages

The relationship between ACL and severity of BC patients was further investigated. With the progression of the disease, the AC of CD3^+^, CD4^+^, CD8^+^, B, and NK cells showed varying degrees of decline (Figure 2). The CD3^+^AC in patients at stage IV was lower than that in patients at stages I and II (*P* < 0.001), whereas BC patients at stage III were not significantly different from that in BC patients at stages I and II (Figure 2(a)). The decline of CD4^+^AC was particularly significant in BC patients. Compared with that in BC patients at stages I, II, and III, the CD4^+^AC in BC patients at stage IV decreased most strikingly (*P* < 0.001), which was followed by stage III (*P* < 0.01), stage II (*P* < 0.01), and stage I (*P* < 0.001) (Figure 2(b)). Compared with BC patients at stage I, the CD8^+^AC decreased in BC patients at stage II (*P* < 0.05) and stage III-IV (*P* < 0.01) (Figure 2(c)). Compared with BC patients at stage I, the B AC decreased in BC patients at stage IV (*P* < 0.01) (Figure 2(d)). In addition, the difference in AC of NK cells was only found in BC patients at stages II and IV (*P* < 0.001) (Figure 2(e)). These results suggested that the decrease of CD4^+^ and CD8^+^AC was closely related to different clinical stages; that is, CD4^+^ and CD8^+^AC declined with the exacerbation of BC.

### 3.4. Differences in ACL between the Response and Nonresponse Groups

To further elucidate the relationship between ACL and the curative effect, we divided the BC patients into two groups according to curative effect, namely, response (*R*) group and nonresponse (NR) group. The results revealed that AC of CD3^+^, CD4^+^, CD8^+^, B, and NK cells in the *R* group was significantly higher than that in the NR group (Figure 3). In brief, the results indicate that the higher the ACL, the better the efficacy.

### 3.5. The Accuracy of ACL in the Efficacy Evaluation

To further clarify the accuracy of ACL in determining efficacy, ROC curve analysis was conducted. The ROC curve showed that CD4^+^AC had the highest prediction accuracy. When the Youden index reached a maximum of 0.662, the area under the curve of CD4^+^AC was 0.90 (95% CI 0.859–0.940), the optimal cutoff value of CD4^+^AC was 468.5 cells/*μ*L, and the sensitivity and specificity were 80.9% and 85.3%, respectively. The results suggested that CD4^+^AC can be used as an index to predict the curative effect (Figure 4).

### 3.6. Correlation between CD4^+^AC and the Clinicopathological Parameters of BC

To further analyze the correlation between CD4^+^AC and clinicopathological parameters, we used the median of CD4^+^AC (451 cells/*μ*L) as the cutoff value and divided 237 BC patients into low level (<451 cells/*μ*L) (118 cases) and high level (<451 cells/*μ*L) (119 cases. The results showed that family history, previous medical history, pathological category, clinical stages, lymphatic metastasis, distant metastases, vessel carcinoma embolus, and treatments were significantly correlated with the CD4^+^ level (*P* < 0.05), whereas age, age of menarche, menopause, tumor size, and differentiation degree were not correlated with the CD4^+^ level (*P* > 0.05) (Table 2).

### 3.7. Effect of ACL on Progression-Free Survival of BC Patients

To investigate the factors influencing PFS in BC patients, we performed univariate and multivariate Cox proportional hazards regression. Analysis showed that the median PFS was 13.57 (range, 2–34) months (Table 3). The univariate analysis suggested that 13 clinicopathological parameters constituted important influencing factors of PFS, including CD4^+^AC, CD8^+^AC, B AC, and NK AC (Table 3). Multivariate analysis revealed that clinical stages (HR = 5.543, 95% CI 1.845–16.650, *P*=0.002) and distant metastasis (HR = 1.852, 95% CI 1.078–3.180, *P*=0.026) contributed to unfavorable prognostic factors, whereas CD4^+^AC ≥ 451 cells/*μ*L (HR = 0.431, 95% CI 0.267–0.697, *P*=0.001) and CD8^+^AC ≥ 324 cells/*μ*L (HR = 0.623, 95% CI 0.426–0.913, *P*=0.015) contributed to favorable prognostic factors (Table 3 and Figure 5). The correlation between ACL and PFS was assessed by Kaplan–Meier survival curves, as shown in Figure 6. In the log-rank test, the median PFS in groups with CD4^+^AC < 451 cells/*μ*L, B AC < 155 cells/*μ*L, and NK AC < 162 cells/*μ*L was 7 months, 11 months, and 10 months, respectively, while in group with CD4^+^AC ≥ 451 cells/*μ*L, B AC ≥ 155 cells/*μ*L, and NK AC ≥ 162 cells/*μ*L, the median PFS was not reached (*P* < 0.001) (Figures 6(b), 6(d), 6(e)). The median PFS in groups with CD8^+^AC < 324 cells/*μ*L was 11 months, and in groups with CD8^+^AC ≥ 324 cells/*μ*L, the median PFS was 26 months (*P*=0.001) (Figure 6(c)). Remarkably, CD3^+^AC had hardly any effect on PFS (Figure 6(a)).

## 4. Discussion

The study showed that it was convenient and accurate to apply the single-platform flow cytometry to analyze the PL and ACL in BC patients. Currently, the PL is most commonly used to evaluate the immune function of tumor patients in clinical practice, whereas the detection of ACL is relatively insufficient, which may lead to a neglect of serious impairment of the immune function of cancer patients. The percentage of lymphocyte subsets represents the composition and proportion of lymphocytes, and reflects the development and differentiation ability of lymphocytes, whereas the absolute counts of lymphocyte subsets represent the number of lymphocytes and reflects the proliferation ability of lymphocytes [21]. At present, there are some controversies in evaluating the immune status and prognosis of tumor patients by the percentage of lymphocyte subsets. Studies have found [22] that the percentage of CD3^+^, CD4^+^, CD4^+^/CD8^+^, and NK cells in peripheral blood of NSCLC patients with stage IV was negatively correlated with the number of circulating tumor cells. A study [23] showed that NSCLC patients had higher baseline percentages of CD3^+^, CD4^+^, and CD8^+^ cell, while lower percentages of NK cell had longer OS. In contrast, another study [24] found that neither the percentage of CD8^+^, CD19^+^, and CD56^+^ lymphocyte subsets nor the CD4^+^/CD8^+^ ratio in peripheral blood was significant predictors or prognostic factors in patients with metastatic breast cancer. The percentage of lymphocyte subsets has some uncertainties in evaluating the immune status and prognosis of patients. Therefore, in recent years, more and more researchers have used the absolute count of lymphocyte subsets as an important immune indicator for the prognosis and efficacy of tumor patients.

The immune system, as a line of defense of the human body against the invasion of pathogens and malignant tumors, consists of cellular immunity and humoral immunity. Studies have shown that cellular immunity plays a vital role in the process of antitumor immunity [25, 26]. The CD3^+^T, as a major in the process of cellular immunity, mainly consists of CD4^+^T and CD8^+^T. The CD4^+^T, playing an immune-modulating role, can assist the B cells to produce antibodies and in the meantime secrete cytokines to enhance the CD8^+^*T* to kill tumors [27]. CD4^+^ helps to initiate a gene expression program of CD8^+^ via multiple molecular mechanisms to enhance the function of CD8^+^CTLs and overcome the obstacle of antitumor immunity [28]. Thus, the CD4^+^T can target tumor cells in various ways, either directly by eliminating tumor cells through the cytolytic mechanism or indirectly by modulating the tumor microenvironment [29]. The increase in the number of CD4^+^T indicates that the immune response is improved and the antitumor activity is reinforced [30]. The CD8^+^T can be classified into cytotoxic T lymphocytes (CTLs) and inhibitory cells. CTLs, as a preferred tool to target tumors, can detect extracellular antigens presented by MHC class I molecules expressed by all tumor cell types [31]. B cells, whose surface marker is CD19^+^, are mainly involved in humoral immunity, and thus, its expression level can be used to evaluate the strength of humoral immunity [32]. NK cells, expressing a specific marker of CD16^+^ or CD56^+^, are a group of cells with special properties and do not have antigen-recognition receptors on the surface [33]. NK cells are the immune cells first activated in the antitumor immunity and important cytotoxic cells in the innate immunity, which can be activated and then perform their effector functions without antigenic stimulation [34]. The decreased number of NK cells indicates that the immune system becomes less capable of monitoring, killing, and clearing tumor cells [35, 36]. Therefore, the detection of the ACL in tumor patients is of great significance for understanding the changes of patients' condition and prognosis [37, 38].

Our study suggested that ACL can be served as a potential biomarker of peripheral blood immune impairment in BC patients to monitor the immune function and to predict the prognosis and therapeutic effects. It is the first of its kind to report the clinical value of peripheral ACL in BC patients for prognosis, despite that some studies claimed that the total number of peripheral blood lymphocytes was associated with the prognosis and therapeutic effects [14, 15, 19, 39, 40]. Our study has made the following findings. Firstly, there was no significant difference in the percentages of CD3^+^, CD4^+^, CD8^+^, B, and NK cells between NCs and BC patients. However, the AC of CD3^+^, CD4^+^, CD8^+^, B, and NK cells decreased markedly in BC patients compared to that in NCs. This finding sheds some light on the necessity and importance of detecting ACL in BC patients in addition to the percentage. This may help us to understand the immunologic injury of BC patients, analyze the clinical condition, and predict the curative effect [11]. Secondly, CD4^+^ had a close negative correlation to clinical stages and thus decreased with the development and deterioration of BC. Compared with that in BC patients at stages I and II, the CD4^+^AC in BC patients at stages III and IV decreased more significantly. Compared with BC patients at stage I, the CD8^+^AC decreased in BC patients at stages II, III, and IV, too. Interestingly, ACL were positively correlated with curative effect. In patients in the response group, AC of CD3^+^, CD4^+^, CD8^+^, B, and NK cells were significantly higher than that in patients in the nonresponse group. Finally, our study reveals that BC patients with CD4^+^AC ≥451 cells/*μ*L or CD8^+^AC ≥324 cells/L demonstrated a longer PFS than BC patients with CD4^+^AC <451 cells/*μ*L or CD8^+^AC <324 cells/*μ*L, which is consistent with our previous study [41]. This indicates that more attention should be paid to CD4^+^ and CD8^+^AC in the antitumor immunity.

The increased number of CD4^+^ and CD8^+^ can signify a good prognosis in BC patients, which is consistent with previous studies [42, 43]. CD4^+^T can promote the activation of CD8^+^CTLs, boost the effector and memory functions of CTLs, and reduce the immunosuppression of CTLs, which helps T cells amplify their response to tumor-associated antigens without generating an autoimmune response [44]. Additionally, the specific binding of antigen to CD4^+^ can enable the dendritic cells to optimize antigen presentation and deliver cytokines and costimulation signals specific to CD8^+^, eventually promoting their cloning, amplification, and differentiation into effector or memory T cells [45]. In brief, the low ACL in BC patients indicates that the immune function of patients is impaired. The patient's impaired immune system could not stop the tumor from progressing [46]. Thus, it is essential to enhance the immune function of BC patients and improve their antitumor ability during the treatment.

Consequently, as the ACL not only reflects the immune status of the body but also can be used to predict disease prognosis and the curative effect, more attention should be paid to the changes of the ACL in clinical practice to provide more referential values to predict the patient's condition and prognosis in clinical treatment.

Our study has some limitations. Firstly, this study is a retrospective study with a relatively small sample size, so some important prognostic factors were not included in the analysis, which may cause some information bias. Secondly, all data included in the study were from a single center. Multicenter studies with large sample sizes are needed to generalize our findings.

## 5. Conclusions

This study shows that it was ACL, rather than PL, that was severely impaired in BC patients, which was correlated to the progression of the tumor, PFS, and efficacy in clinical treatment. Thus, it is necessary and pivotal to detect ACL in clinical practice. In a nutshell, our study suggests that ACL can be used as a potential peripheral blood biomarker for monitor immune impairment and predicting the prognosis and therapeutic effect of BC patients.

## Figures and Tables

**Figure 1:** Comparison of percentages and absolute counts of lymphocyte subsets between BC patients and NCs. (a) The comparison of percentages of lymphocyte subsets between BC patients and NCs. (b) The comparison of the absolute counts of lymphocyte subsets between BC patients and NCs. (c) and (e) show the comparison of percentages of lymphocyte subsets between BC patients at different stages and NCs. (d) and (f) show the comparison of the absolute counts of lymphocyte subsets between BC patients at different stages and NCs. BC, breast cancer; NCs, normal controls; ^*∗∗∗*^*P* < 0.001.

**Figure 2:** Comparison of ACL in BC patients at different clinical stages. AC of CD3^+^ (a) CD3+CD4+ (b) CD3+CD8+ (c) B cells (d) and NK cells (e) in BC patients at different stages. AC, absolute count; ACL, absolute count of lymphocyte subsets; ^*∗*^*P* < 0.05; ^*∗∗*^*P* < 0.01; ^*∗∗∗*^*P* < 0.001.

**Figure 3:** Comparison of ACL between the response and nonresponse groups. CD3^+^AC (a) CD4+AC (b) CD8+AC (c) B AC (d) and NK AC (e) in the response and nonresponse groups. AC, absolute count; R response; NR, nonresponse. ^*∗*^*P* < 0.05; ^*∗∗*^*P* < 0.01; ^*∗∗∗*^*P* < 0.001.

**Figure 4:** ROC curves analysis predicting efficacy using ACL. ROC, receiver operating characteristic curve; AC, absolute count; ACL, absolute count of lymphocyte subsets.

**Figure 5:** The forest plots of factors affecting the progression-free survival. OR > 1 indicates that the variable is considered a risk factor. OR < 1 represents that the variable is considered a protective factor. The bolded value represents that the *P* value was significant.

**Figure 6:** The Kaplan–Meier curve of PFS for BC patients with high or low absolute count of CD3^+^ (a) CD4^+^ (b) CD8^+^ (c) B (d) and NK cells (e) BC, breast cancer; AC, absolute count.

**Table 1:** Clinicopathological characteristics of 237 breast cancer patients.

Characteristics	N	%
Age		
≥64	113	47.7
<64	124	52.3

Family history		
Yes	116	48.9
No	121	51.1

Previous medical history		
Yes	199	84.0
No	38	16.0

Age of menarche		
<12	121	51.1
≥12	116	48.9

Menopause		
Yes	208	87.8
No	29	12.2

Tumor size		
<2 cm	61	25.7
2-5 cm	127	53.6
>5 cm	49	20.7

Pathological category		
ILC	28	11.8
IDC	209	88.2

Differentiation		
High	56	23.6
Medium/low	181	76.4

Clinical stages		
I + II	89	37.6
III + IV	148	63.4

Lymph node metastasis		
Yes	158	66.7
No	79	33.3

Distant metastasis		
Yes	117	49.4
No	120	50.6

Vessel carcinoma embolus		
Yes	59	21.6
No	178	78.4

Treatments		
Surgery	83	35.0
Surgery + chemotherapy	82	34.6
Surgery + endocrinotherapy	72	30.4

Notes: ILC, invasive lobular carcinomas; IDC, invasive ductal carcinoma.

**Table 2:** Relationship between CD4^+^AC and clinicopathological parameters of breast cancer patients.

Characteristics	Low level	High level	*χ* ^2^	*P* value
	<451 cells/*μ*L	≥451 cells/*μ*L		
Age			3.072	0.08
<64	63	50		
≥64	55	69		

Family history			7.089	0.008
Yes	68	48		
No	50	71		

Previous medical history			4.393	0.036
Yes	105	94		
No	13	25		

Age of menarche			1.217	0.27
<12	56	65		
≥12	62	54		

Menopause			1.031	0.31
Yes	101	107		
No	17	12		

Tumor size			1.016	0.602
<2 cm	27	34		
2-5 cm	66	61		
>5 cm	25	24		

Pathological category			10.215	0.001
ILC	6	22		
IDC	112	97		

Differentiation			0.777	0.378
High	25	31		
Medium/low	93	88		

Clinical stages			57.692	<0.001
I + II	16	73		
III + IV	102	46		

Lymph node metastasis			34.566	<0.001
Yes	100	58		
No	18	61		

Distant metastasis			48.305	<0.001
Yes	85	32		
No	33	87		

Vessel carcinoma embolus			28.04	<0.001
Yes	47	12		
No	71	107		

Treatments			22.069	<0.001
Surgery	42	41		
Surgery + chemotherapy	55	27		
Surgery + endocrinotherapy	21	51		

Notes: ILC, invasive lobular carcinomas; IDC, invasive ductal carcinoma.

**Table 3:** Univariate and multivariate analysis of prognostic factors of PFS.

Characteristics		Univariate		Multivariate	
		HR (95% CI)	*P* value	HR (95% CI)	*P* value
Age	<64	1 [reference]	0.583		
	≥64	0.908 (0.642–1.282)			

Family history	No	1 [reference]	<0.001	1.106 (0.760–1.609)	0.600
	Yes	1.969 (1.384–2.801)			

Previous medical history	No	1 [reference]	0.002	1.064 (0.552–2.050)	0.854
	Yes	2.667 (1.436–4.953)			

Smoking	No	1 [reference]	0.051		
	Yes	1.511 (0.999–2.285)			

Drink	No	1 [reference]	0.835		
	Yes	0.952 (0.602–1.507)			

Age of menarche	<12	1 [reference]	0.027	1.019 (0.709–1.466)	0.917
	≥12	1.482 (1.046–2.101)			

Menopause	No	1 [reference]	0.301		
	Yes	1.368 (0.775–2.480)			

Tumor size	<2 cm	1 [reference]	0.014	0.960 (0.606–1.520)	0.861
	≥2 cm	1.716 (1.115–2.640)			

Pathological category	ILC	1 [reference]	0.004	0.599 (0.273–1.316)	0.202
	IDC	2.834 (1.381–5.813)			

ER	Negative	1 [reference]	0.198		
	Positive	0.796 (0.562–1.127)			

PR	Negative	1 [reference]	0.350		
	Positive	0.848 (0.599–1.199)			

Her2	Negative	1 [reference]	0.979		
	Positive	1.005 (0.694–1.456)			

Differentiation	High	1 [reference]	0.263		
	Medium/low	1.271 (0.835–1.934)			

Clinical stages	I + II	1 [reference]	<0.001	5.543 (1.845–16.650)	0.002
	III + IV	15.425 (7.796–30.521)			

Lymphatic metastasis	No	1 [reference]	<0.001	1.307 (0.486–3.521)	0.596
	Yes	10.563 (5.516–20.228)			

Distant metastasis	No	1 [reference]	<0.001	1.852 (1.078–3.180)	0.026
	Yes	7.497 (4.856–11.572)			

Vessel carcinoma embolus	No	1 [reference]	<0.001	1.425 (0.953–2.131)	0.143
	Yes	3.797 (2.642–5.457)			

Treatment	Surgery	1 [reference]	0.403		
	Surgery + chemotherapy	0.840 (0.559–1.263)			
	Surgery + endocrinotherapy	0.748 (0.486–1.151)	0.186		

CD3^+^AC (cells/*μ*L)	<924	1 [reference]	0.862		
	≥924	1.031 (0.730–1.457)			

CD4^+^AC (cells/*μ*L)	<451	1 [reference]	<0.001	0.431 (0.267–0.697)	0.001
	≥451	0.170 (0.112–0.257)			

CD8^+^AC (cells/*μ*L)	<324	1 [reference]	0.001	0.623 (0.426–0.913)	0.015
	≥324	0.548 (0.385–0.781)			

B AC (cells/*μ*L)	<155	1 [reference]	<0.001	0.955 (0.644–1.415)	0.817
	≥155	0.493 (0.345–0.703)			

NK AC (cells/*μ*L)	<162	1 [reference]	<0.001	1.021 (0.677–1.539)	0.922
	≥162	0.425 (0.295–0.611)			

Notes: AC, absolute count; ER, estrogen receptor; PR, progesterone receptor; Her2, human epidermal growth factor receptor 2.

## Data Availability

The datasets used and/or analyzed during the current study are available from the corresponding author upon reasonable request.
